This article has been retracted.

# Effects of Aidi injection on life quality and incidence of adverse reactions in patients with non-small cell lung cancer compared with traditional chemotherapy: a systematic review and meta-analysis

**DOI:** 10.3389/fonc.2023.1145029

**Published:** 2023-04-28

**Authors:** Qing Fang, Biyun Yu, Hui Xu, Yuanyuan Xu

**Affiliations:** Department of Pulmonary and Critical Care Medicine, Ningbo Medical Center Lihuili Hospital, Ningbo, China

**Keywords:** Aidi injection, traditional chemotherapy, NSCLC, life quality, incidence of adverse reactions

## Abstract

**Objective:**

Although the clinical application value of Aidi injection when treating non-small cell lung cancer (NSCLC) patients is explained only by the effectiveness of a certain literature or the improvement of a certain evaluation index, and the result is not convincing. To evaluate the effect of Aidi injection on life quality and incidence of adverse reactions in patients with NSCLCcompared with traditional chemotherapy.

**Methods:**

PubMed, EMBASE, ScienceDirect, Cochrane Library, China Journal full-text Database (CNKI), VIP full-text Database, Wanfang Database and Chinese Biomedical Literature data (CBM), search relevant Chinese and foreign periodicals, conference papers, degree papers, etc. were searched Database and China Biomedical Literature Database (CBM) to search case-control trials of Aidi injection when treating NSCLC patients. The retrieval period begins with the establishment of the database and ends when the database is closed. Cochrane Handbook 5.3 was adopted to assess the bias risk of each contained literature based on independently extracted data by two researchers. A meta-analysis of the collected data was carried out using RevMan5.3 statistical software.

**Results:**

2306 articles were retrieved by computer database, 1422 articles were harvested by excluding repeated studies, 865 articles were harvested by preliminary reading of article titles and abstracts, and 533 articles were initially contained by excluding unrelated studies, reviews, case reports and uncontrolled articles, and then the full text of the literature was carefully read. Eight clinical controlled studies were finally included, with a total of 784 samples, after excluding 525 literatures with incomplete data and no primary outcome indicators. Data from the contained studies were not noticeably heterogeneous in the meta-analysis of treatment effectiveness. The fixed effect model analysis indicated that the treatment effective rate of the study group was noticeably better, and the difference was statistically significant(P<0.05). The findings of the heterogeneity test were clearly heterogeneous among the contained research data, according to the meta-analysis of the levels of T lymphocyte subsets following treatment. The random effect model analysis indicated that the improvement of the cellular immune function of the research group was obvious, and the difference was statistically significant (P<0.05). According to the meta-analysis of the life quality scores after treatment, data from the contained research were evidently heterogeneous, according to results of the heterogeneity test. The random effect model analysis indicated that the life quality of the study group was noticeably higher, and the difference was statistically significant (P<0.05). The levels of serum vascular endothelial growth factor (VEGF) after treatment were measured by meta. Data from the contained research were evidently heterogeneous, according to results of the heterogeneity test. Random effect model analysis indicated that the level of serum VEGF in the study group was noticeably lower, and the difference was not statistically significant (P>0.05). A meta-analysis was conducted on the incidence of adverse reactions after treatment. The results of the heterogeneity test indicated that data from the contained research were evidently heterogeneous. The incidence was noticeably lower, and the difference was statistically significant (P<0.05). The funnel chart was drawn based on the effective rate of treatment, the level of T lymphocyte subsets, the score of life quality, the level of serum VEGF and the incidence of adverse reactions, and the publication bias analysis was carried out. The results indicated that most of the funnel maps were symmetrical and a small part of them were asymmetrical, suggesting that despite the heterogeneity of the study and the small number of included literatures, a publication bias was apparent in the included literature.

**Conclusion:**

Based on routine chemotherapy associated with Aidi injection, the therapeutic effect of NSCLC patients can be noticeably enhanced, the effective rate of treatment can be noticeably promoted, the immune function and life quality can be improved, and the incidence of adverse reactions is low, which is worth popularizing in clinical practice, but several studies and follow-ups are needed to improve methodological quality and to verify the results over a longer period of time.

## 1 Introduction

Bronchogenic carcinoma (lung cancer for short) is a malignant tumor originating from bronchial mucosa or gland. It is one of the most obvious malignant tumors. Its morbidity and mortality are increasing all over the world. There are more than 600,000 new cases of lung cancer in China every year, and its morbidity and mortality rank first among many cancers (1–3). It is estimated that 80 percent of lung cancers are non-small cell lung cancers (NSCLCs). Surgical treatment is the most common treatment for lung cancer at an early stage. Furthermore, because of the latent onset of NSCLC in the early stage, when patients are diagnosed, they are usually in the middle or late stages, so surgery cannot be conducted, and radiotherapy and chemotherapy cannot be administered. Toxic and side effects are more common (4). In the United States, only 16.8% of patients diagnosed with lung cancer survive for more than 5 years, and this proportion is even lower in developing countries (5). Therefore, how to make patients receive reasonable treatment, improve the treatment effect, and improve the prognosis is particularly important when treating lung cancer clinically.

The aim of the treatment of advanced malignant tumors is not only to prolong the survival time of patients, but also to prolong the survival time and improve the life quality at the same time. There are unique advantages to traditional Chinese medicine (TCM) when it comes to reducing symptoms and improving life quality. In clinic, TCM and integrated traditional Chinese and western medicine have certain characteristics and advantages when treating lung cancer, especially in the clinical treatment of lung cancer (5). Aidi injection is a unique compound injection refined from TCM. The active ingredients are ginseng, astragalus, Acanthopanax senticosus and Mylabris (6). Ginseng: sweet, slightly bitter, lukewarm, heart, lung and spleen meridians, with the effects of invigorating vital energy, tonifying the spleen and lung, invigorating the nerves, astragalus sweet, lukewarm, returning to the spleen and lung meridians, replenishing qi and yang, tonifying the body, promoting water and reducing swelling, supporting sore and promoting muscle; Acanthopanax senticosus: Xin, bitter, warm, liver and kidney meridians, with the effect of dispelling rheumatism, strengthening muscles and bones, and diuresis. Mylabris: Xin, warm, toxic, return to the liver, kidney and stomach, with the effect of breaking blood stasis, attacking poison and dispersing knots. All kinds of medicines are used together to play the function of replenishing qi and promoting fluid, calming the mind, removing blood stasis and attacking toxin (7–9). Modern pharmacological studies have confirmed (10) that ginseng can inhibit the formation of new blood vessels around tumors and the proliferation of vascular endothelial cells, promote tumor cell apoptosis, enhance the phagocytosis and killing functions of macrophages and natural killer cells (NK), and improve immunity. It has a wide range of anti-tumor effects; astragalus polysaccharides can enhance human immunity, increase white blood cells, enhance thymus dependent lymphocytes (T-lymphocytes), lymphokine activated killer cells (LAK), NK activity, the effect of Pl; the glycosides and the polysaccharides in the extract of Acanthopanax senticosus can induce the production of interferon-y and improve the activity of recombinant human tumor necrosis factor-β (TNF-β) and NK cells in the peripheral blood of lung cancer. Cantharidin, the main component of cantharidin, can inhibit the metabolism of cancer cells and induce tumor cell apoptosis. Aidi injection organically integrates the active components of the above-mentioned TCM according to a certain proportion, acts on tumor cells and tissues with multiple targets, regulates the immune function of the body, and gives full play to the biological synergism of various effective components.

The clinical application value of Aidi injection when treating NSCLC patients is explained only by the effectiveness of a certain literature or the improvement of a certain evaluation index, and the result is not convincing. High-quality research evidence is still needed to support it (4). In this context, further related research is very necessary, we need to testify the therapeutic effect of Aidi injection on patients with NSCLC through more and more authoritative scientific research, in order to provide a theoretical basis for the promotion and application of this treatment. Therefore, this study makes a systematic, quantitative and comprehensive analysis of the results of similar independent studies through Meta analysis, in order to evaluate the effect of Aidi injection compared with traditional chemotherapy on the life quality and the incidence of adverse reactions in patients with NSCLC, and to offer objective basis for its clinical application and further research.

## 2 Research contents and methods

### 2.1 The sources and retrieval methods of documents

Literature search was conducted with free words + subject words, with the key words of Aidi injection; traditional chemotherapy; NSCLC; life quality; incidence of adverse reactions; meta-analysis; Aidi injection; Traditional chemotherapy; NSCLC; Life quality; Incidence of adverse reactions; Meta analysis et al., from January 2010 to April 2022.PubMed, EMBASE, ScienceDirect, Cochrane Library, China Journal full-text Database (CNKI), VIP full-text Database, Wanfang Database and Chinese Biomedical Literature data (CBM), search relevant Chinese and foreign periodicals, conference papers, degree papers, etc.were searched Database and China Biomedical Literature Database (CBM) to search case-control trials of Aidi injection when treating NSCLC patients.

### 2.2 Literature inclusion criteria and exclusion criteria

#### 2.2.1 Literature inclusion criteria

(1) Type of study: all the clinical controlled trials in which Aidi injection was adopted when treating NSCLC patients; (2) subjects: patients with NSCLC diagnosed by pathological biopsy or immunohistochemistry were diagnosed with NSCLC according to the relevant literature (11), the performance status (PS) score of the patients was 2[The patient is capable of walking and self-care, but has lost the ability to work and is able to get up and move for at least half of the day (in other words, the patient needs to be in bed for part of the day)], the expected survival time was more than 3 months, at least one lesion was ≥ 1cm; (3) There are no contraindications to chemotherapy before treatment, and there are no obvious abnormalities in liver and kidney function, hematology, and electrocardiogram.; (4) Karl Fischer score ≥ 60 points or ECOG score of 0-2 points (The patient can take care of himself with the help of others.); (5) All the patients have not received chemotherapy before treatment; (6) The total size of subjects is more than 50 (According to the sample size of screening after reading the literature abstract).

#### 2.2.2 Literature exclusion standard

(1) It is not a case-control study; (2) it is impossible to use the data because the report is incomplete; (3) the research content should be repeated, and the latest research taken into consideration; (4) study findings did not indicate that the study had a curative effect; (5) Review of related literature; (6) Accompanied by serious internal medicine diseases and infections; (7) Accompanied by other malignant tumors; (8) Lung cancer is a metastasis of other tumors.

### 2.3 Quality evaluation and data extraction

1) Bias risk assessment contained in the study: Based on Cochrane System Review Manual 5.3, a bias risk assessment tool was used to conduct the evaluation.

2) Literature screening and data extraction: Independently, two researchers screened literature, gathered data, assessed quality, and cross-checked results. A disagreement should be discussed and resolved, or a third researcher should be invited to contribute to the judgement. A document management system called Note Express was adopted, along with an office program called Excel, to manage and extract research data. In case the literature includes incomplete data, contact the author for additions. The contents of data extraction include (1) Basic information: Author, publication time, number of cases; (2) Intervention measures: Scheme, course of treatment; (3) Outcome indicators: Effective rate of treatment, level of T lymphocyte subsets, life quality, serum VEGF level, incidence of adverse reactions.

### 2.4 Statistical processing

Meta analysis was conducted using RevMan5.3 software. Counting data was indexed by relative risk (OR) and measurement data was indexed by mean difference (MD). The point estimate and 95% confidence interval (CI) of each effect are given. χ 2 test was adopted for heterogeneity test, and I^2^ was adopted to judge the heterogeneity. Fixed effect models are adopted if there exhibits no heterogeneity; if there exhibits heterogeneity, subgroup, sensitivity, or descriptive analysis are adopted, and the random effect model is adopted if there exhibits heterogeneity. The difference exhibited statistically noticeable, and the difference was statistically significant(P<0.05). The inverted funnel chart was further drawn to analyze the publication bias contained in the literature. Eggers’s test is adopted to check the asymmetry of the funnel chart. Whenever the p value of this test is less than 0.1, the TrimandFill method can be used to correct the funnel chart and adjust the effect of the potential release deviation. The reason for using the fixed model was the situation where the heterogeneity between the observed results is low.

## 3 Results and analysis

### 3.1 The results of literature retrieval and the basic situation of literature inclusion

2306 articles were retrieved by computer database, 1422 articles were harvested by excluding repeated studies, 865 articles were harvested by preliminary reading of article titles and abstracts, and 533 articles were initially contained by excluding unrelated studies, reviews, case reports and uncontrolled articles, and then the full text of the literature was carefully read. A total of 784 samples were included in the final analysis from 8 clinical controlled studies (12–19), which included 525 literatures with incomplete data and no primary outcome indicators. **Figure 1** depicts the screening diagram for the literature (Reason 1: 188 with duplicate documents; Reason 2: 150 with other chemotherapy; Reason 3: 179 with statements and others (The article explicitly states that data sharing is not allowed).), and **Table 1** summarizes the basic characteristics of the contained literature.

**Figure 1:** Literature screening diagram. "*" means Articles searched from Database. "**" means Duplicate article.

**Table 1:** Basic characteristics of literature.

Include the literature	Year of publication	N (C/T)	Intervention method		Outcome index	Research type	Grouping method	Blind or not
			C	T				
Cao Jianzhong (12)	2020	40/41	CAP Scheme	CAP Plan + Eddie	(1)(2)(5)	Prospective study	Random grouping	No
Xiong Xuefang (13)	2021	48/48	TP Scheme	TP Plan + Eddie	(1)(2)(3)(4)(5)	Prospective study	Simple digital table method	No
Han Ruili (14)	2015	36/36	GP Scheme	GP Plan + Eddie	(1)(2)(3)(5)	Prospective study	Random grouping	No
Ma Yanhua (15)	2020	67/65	GC Scheme	GC Plan + Eddie	(1)(3)(5)	Prospective study	Random grouping	No
Liu Huafeng (16)	2019	44/44	GP Scheme	GP Plan + Eddie	(1)(2)(4)	Prospective study	Simple digital table method	No
Shen Wenming (17)	2022	60/60	Docetaxel + cisplatin	Docetaxel + cisplatin + Eddie	(1)(4)	Prospective study	Simple digital table method	No
Su Shujuan (18)	2017	40/39	Gemcitabine + cisplatin	Gemcitabine + cisplatin + Eddie	(1)(2)(5)	Prospective study	Simple digital table method	No
Zhou Dongmei (19)	2018	58/58	GP Scheme	GP Plan + Eddie	(1)(3)(5)	Prospective study	Random grouping	No

C, control group; T, research group; CAP, cyclophosphamide + doxorubicin + cisplatin; TP, Paclitaxel and cisplatin; GP/GC, gemcitabine + cisplatin; Random grouping: A method of randomly assigning research subjects to experimental and control groups. Simple digital table method: Simple digital table method also known as the random number table method, which is a method of using a random number table to draw samples; (1) Treatment effective rate; (2) T lymphocyte subsets; (3) Life quality score; (4) Serum VEGF level; (5) Incidence of adverse reactions.

### 3.2 Evaluation of the quality of the methodology contained in the literature

(1) Random allocation method: All literatures describe the random method in detail. Because of the objective nature of the random allocation method, the risk is low.; (2) Allocation hiding: All literature does not mention whether the allocation is hidden or not, so it is defined as risk uncertainty; (3) Blind method: The blind method is not mentioned in all the literature, so the performance risk is defined as high risk and the detection risk is defined as low risk; (4) Data integrity: All the literature reports are complete, there is no missing case data, which is a low risk; (5) Selective report: None of the literature has harvested its trial plan, so it is classified as risk uncertainty; (6) Other biases: Some literature reports found other risks, which are high risk. The risk bias analysis is indicated in **Figures 2**, **3**.

**Figure 2:** Risk bias chart.

**Figure 3:** Summary chart of risk bias.

### 3.3 Meta analysis result

#### 3.3.1 Treatment effective rate

Treatment effective rate is the frequency of treatment effectiveness in patients receiving treatment. Total effective rate = cure rate + apparent efficiency + effective rate. Total effective rate % = (effective + effective)/number of patient cases× 100% There were 8 clinical controlled studies contained in this study, with 784 samples. Meta-analysis was conducted on the treatment effective rate. The results of the heterogeneity test indicated that Chi^2 = ^2.78, df=6, P=0.84, I^2 = ^0%, the results indicated that data from the contained research were evidently heterogeneous. According to the analysis of fixed effect model (**Figure 4**), the effective rate of the study group was noticeably better, and the difference was statistically significant(P<0.05).

**Figure 4:** Forest analysis map of the comparison of treatment efficiency. Odds ratio (OR) is a way of describing probability; M-H, Mantel-Haenszel.

#### 3.3.2 T lymphocyte subsets level

As the **Figure 5** reported, this study contained 8 clinical control studies with a total of 784 samples, the levels of T lymphocyte subsets after treatment were measured by Meta. The results of heterogeneity test indicated that Chi^2 = ^1251.93, df=18 P<0.00001, I^2 = ^99%, the results indicated that data from the contained research were evidently heterogeneous. The random effect model analysis indicated that the improvement of cellular immune function in the study group was noticeably better, and the difference was statistically significant(P<0.05).

**Figure 5:** Forest analysis map of comparison of T lymphocyte subsets after treatment. IV, Inverse variance.

#### 3.3.3 Life quality score

As the **Figure 6** reported, there were 8 clinical controlled studies contained in this study, with 784 samples. Meta-analysis was conducted on the life quality scores after treatment. The results of the heterogeneity test indicated that Chi^2 = ^1731.83, df=17, P<0.00001, I^2 = ^99%, the results indicated that data from the contained research were evidently heterogeneous. The random effect model analysis indicated that the life quality in the study group was noticeably higher after treatment, and the difference was statistically significant(P<0.05).

**Figure 6:** Forest analysis map of comparison of life quality scores.

#### 3.3.4 Serum vascular endothelial growth factor level

As the **Figure 7** reported, this study contained 8 clinical control studies with a total of 784 samples. The serum VEGF levels after treatment were measured by meta. The results of heterogeneity test indicated that Chi^2 = ^16.44, df=2, P=0.0003, I^2 = ^88%, the results indicated that data from the contained research were evidently heterogeneous, and the random effect model analysis indicated that the serum VEGF level of the study group was noticeably lower after treatment, and the difference was not statistically significant(P>0.05).

**Figure 7:** comparison of serum VEGF levels after treatment.

#### 3.3.5 Incidence of adverse reactions

As the **Figure 8** reported, there were 8 clinical controlled studies with 784 samples contained in this study. A meta-analysis was conducted on the incidence of adverse reactions after treatment. The adverse reactions mainly contained bone marrow suppression, digestive tract reactions, liver and kidney function damage, and leukopenia, and thrombocytopenia, etc., according to the heterogeneity test results: Chi^2 = ^28.58, df=19, P=0.07, I^2 = ^34%, the results indicated that data from the contained research were evidently heterogeneous, which was measured by fixed effect model (**Figure 8**). Compared with the control group, the incidence of adverse reactions in the study group was noticeably higher, and the difference was statistically significant(P<0.05).

**Figure 8:** Forest map with comparative incidence of adverse reactions.

#### 3.3.6 Publication bias analysis

Funnel charts were drawn on the basis of treatment efficacy, T lymphocyte subsets, life quality score, serum VEGF levels and incidence of adverse reactions, and publication bias was measured (see **Figures 9**–**13**). The results show that most of the funnel charts are symmetrical and a small part of them are asymmetrical, suggesting that there exhibits a certain publication bias in the contained literature. This may be relevant to the heterogeneity of the study and the small number of contained literatures.

**Figure 9:** Funnel chart based on treatment efficiency.

**Figure 10:** Funnel chart based on T lymphocyte subsets after treatment.

**Figure 11:** Funnel chart based on life quality score.

**Figure 12:** Funnel chart based on serum VEGF level after treatment.

**Figure 13:** Funnel chart based on the incidence of adverse reactions.

## 4 Analysis and discussion

In recent years, there are more and more clinical reports on the application of Aidi injection when treating NSCLC, suggesting that Aidi injection has high application value in the clinical treatment of NSCLC patients, but there are great differences between different research designs and a variety of evaluation indicators. At present, the mortality rate of lung cancer ranks first among all cancers in the world, among which NSCLC is the most obvious. In addition to squamous cell carcinomas and large cell carcinomas, adenocarcinomas are also classified as NSCLC. Patients with NSCLC have relatively slow cell growth and division, as well as long timeframes for the spread and metastasis of the cancer compared with patients with small cell carcinoma (20). Patients with NSCLC are often accompanied by symptoms of different severity, such as cough, chest tightness, fever, chest pain, hemoptysis, and loss of appetite. When the disease progresses to the later stage, it will affect other tissues and organs of the patient, making treatment much more difficult, and increase the risk of death. The study found that (21, 22), the mortality rate of NSCLC has exceeded that of breast cancer, prostate cancer and colorectal cancer combined for many years. Chemotherapy is the first choice of treatment, because the chemotherapeutic drugs themselves have strong toxic effects, which will cause some damage to the immune system of patients, reduce their life quality, and cause adverse reactions such as gastrointestinal reactions and myelosuppression (23). Therefore, it is of great significance to find a therapeutic drug which can not only improve the effect of chemotherapy, but also enhance immune function and reduce toxic reaction.

Studies have shown that Aidi injection has pharmacological effects such as inhibiting tumor metastasis, improving patients’ immunity and protecting liver and kidney function, but the reference value of animal test data is limited, which cannot accurately and intuitively reflect the synergistic and attenuating effect of Aidi injection on clinical chemotherapy. Associated with this study, this study finally contained 8 clinical control studies, a total of 784 samples. Meta-analysis of the treatment effective rate revealed that the study group had a noticeably higher treatment effective rate based on fixed effect model analysis, and the difference was statistically significant(P<0.05), which proved that Aidi injection had definite chemotherapeutic synergism, which was consistent with the previous research results. The reason is that Aidi injection contains a variety of TCM ingredients (ginseng, Mylabris, Acanthopanax senticosus and astragalus), among which astragalus can enhance immune function and delay the development of cell senescence; cantharidin is an effective anticancer ingredient. Ginseng has the effects of invigorating fluid, tonifying the spleen and tonifying the lung and calming the nerve. Studies have found that ginseng associated with chemotherapy can enhance the life quality of patients with lung cancer, reduce adverse reactions and noticeably enhance the effect of chemotherapy. Acanthopanax senticosus has the functions of “tonifying essence, strengthening will, strengthening muscles and bones”. The combined use of various medicines can play the effects of eliminating blood stasis and dispersing knots, clearing heat and detoxification, strengthening positive and dispelling pathogenic factors, can treat tumors with multiple targets, and can be used when treating rectal cancer, primary liver cancer, malignant lymphoma, gynecological malignant tumors and lung cancer (24, 25).

Several studies have concluded that immunotherapy attaches importance to NSCLC (26, 27). The development of tumor cells is relevant to the cellular immune function of the body closely, and the two are mutually causal. The use of biomarkers and immune monitoring can help clinicians understand the effects of immunotherapy in patients with NSCLC. The anti-tumor response of the body is mainly a cellular immune response, in which T lymphocytes play a regulatory role in the tumor immune response. The improvement in the number, activity and proportion of CD8+, CD4+ and CD3+ is relevant to the development of tumors closely. Only when the body’s CD4+/CD8+ maintains a normal level, can the normal anti-tumor effect be produced. The meta-analysis of the levels of T lymphocyte subsets after treatment, and the random effect model analysis indicated that the improvement of cellular immune function in the study group was noticeably better, and the difference was statistically significant(P<0.05). The results show that Aidi injection can increase effective rate, improve cellular immune function, improve life quality, reduce serum VEGF level, and reduce incidence of adverse reactions, which is consistent with the results of Xiao Zheng et al. (28). The reason is that ginseng and astragalus in Aidi injection can enhance the function of T cells and B cells, stimulate the production of interferon and interleukin, enhance the activity of LAK cells and NK cells, and then enhance the anticancer effect. Aidi injection can protect the function of T cells, reduce the apoptosis rate of immune cells in patients with advanced NSCLC, increase the positive rate of CD cells, and then inhibit the inhibitory effect of tumor on the immune system.

VEGF is an important part of tumor angiogenesis, which can stimulate the growth and proliferation of vascular endothelial cells, increase vascular permeability and weaken the mechanism of immune response. To a certain extent, it reflects the growth, invasion and metastasis of tumor (29, 30). The serum VEGF levels after treatment were measured by meta, and the random effect model analysis indicated that the serum VEGF level of the study group was noticeably lower, and the difference was not statistically significant(P>0.05). This shows that the treatment of routine chemotherapy associated with Aidi injection can successfully reduce the level of serum VEGF. The reason may be that the four active ingredients in Aidi injection are compatible with each other and complement each other. Among them, Cantharidin can break blood and remove blood stasis, attack toxin and sore, and Radix Astragali can strengthen the root and replenish qi, and Acanthopanax senticosus can benefit qi and invigorate the spleen. It has the effect of tonifying the kidney and calming the nerves. After being refined and made into an injection, it can be used for multi-targeted treatment of tumors, increase the immune function of the body, and can directly kill cancer cells, promote tumor cell apoptosis, and improve the life quality of patients. The meta-analysis of the life quality scores after treatment was carried out, and the random effect model analysis indicated that the life quality of the study group after treatment was noticeably higher, and the difference was statistically significant(P<0.05), which was consistent with the results of previous studies. The main reason why the life quality of the patients in the research group has been greatly improved is that the patient’s condition and physical and mental state have been noticeably improved after the treatment with Aidi injection, and the life quality has naturally improved, enabling them to return to normal life.

In chemotherapy treatment, the toxic and side effects are more harmful to the patient’s body. There are many toxic effects and side effects associated with this drug, including bone marrow suppression, gastrointestinal reactions, and neurological problems. The incidence of adverse reactions is also one of the effective reference indicators to assess the clinical efficacy of cancer patients. A meta-analysis of the incidence of adverse reactions after treatment indicated that the main adverse reactions of patients mainly contained bone marrow suppression, digestive tract reactions, liver and kidney function damage, leukopenia and thrombocytopenia, etc. The incidence of adverse reactions was noticeably higher in the control group, and the difference was statistically significant(P<0.05), indicating that Aidi injection has a satisfactory adjuvant effect in enhancing the life quality and enhancing the tolerance to chemotherapy while improving the clinical efficacy of advanced NSCLC patients. The safety of the treatment is guaranteed, and patients can use it with confidence. The limitations of this study are as follows: (1) the inclusion and exclusion criteria are relatively strict, and the final number of literatures is relatively small; (2) the follow-up time of all studies is not consistent, so there are some limitations, which need to be followed up by scholars to provide more support for the clinical application of Aidi injection in NSCLC patients, and more high-quality case-control trials need to be carried out to verify; (3)The limitations for this study is not following the 2020 version of PRISMA, therefore, the results of this study will be biased;(4)The limitations for this study is this article has not been registered in any of the registry systems, therefore, the results of this study will be biased.

Considering the limitations of this meta-analysis, including heterogeneity, small study size, and inconsistent follow-up time of all studies, possible improvements can be made to existing statistical methods in follow-up studies, such as expanding the time range of literature search, selecting literatures with larger sample size, and limiting the follow-up time of studies, so as to improve the quality and credibility of follow-up studies.

## 5 Conclusion

All in all, it is safe and feasible to combine Aidi injection in combination with Aidi injection in the clinical treatment of NSCLC patients in addition to conventional chemotherapy. AIDI injection can play a synergistic effect, which can significantly improve the quality of life of patients, enhance their immune function, and reduce the occurrence of adverse reactions, which is consistent with the original literature. It can be seen that the treatment plan is worthy of clinical application.

## Data availability statement

The datasets used and/or analyzed during the current study are available from the corresponding author on reasonable request.

## Author contributions

QF contributed to the conception and design of the study. QF acquired the data. QF and BY performed the data analysis and wrote the first draft of the manuscript. HX and YX revised the manuscript critically. All authors contributed to the article and approved the submitted version.
